# Seed Coat Morphology and Sculpturing of Selected Invasive Alien Plants from Lesser Himalaya Pakistan and Their Systematic Implications

**DOI:** 10.1155/2022/8225494

**Published:** 2022-07-25

**Authors:** Farida Anjum, Asif Mir, Yasmeen Shakir, Muhammad Zafar, Shazia Sultana, Maria Ameen, Mushtaq Ahmad

**Affiliations:** ^1^Department of Plant Sciences, Quaid-i-Azam University, Islamabad, Pakistan; ^2^Department of Biochemistry, Hazara University, Mansehra, Pakistan; ^3^Department of Biological Sciences, International Islamic University, Islamabad, Pakistan

## Abstract

Invasive alien species (IAS) are considered as the second major threat to biodiversity after habitat destruction worldwide. They are aggressive competitors and dominate an ecosystem where they introduce and cause reduction in indigenous diversity. Invasive plants alter the evolutionary pathways of native species by competition, niche displacement, hybridization, introgression, predation, and ultimately extinction of native species. Biological invasion also results in economic and environmental damage and harm to human health. Invasive plants have an effective reproductive as well as dispersal mechanisms. Most invasive plants produce abundant fruits and seeds that are widely disseminated and remain viable in the soil for several years. Invasive plants may change their seed character in order to adapt themselves to the new environment and facilitate their performance. A study on seed coat sculpturing in invasive alien plants collected from Lesser Himalaya region, Pakistan, was conducted using scanning electron microscope to determine the importance of seed morphological characters as an additional tool for identification. Quantitative characters such as seed length and width, macromorphological characters including color, hilum position, and seed shape, and micromorphological characters of seed including surface patterns and periclinal and anticlinal wall of seeds were studied. Findings at the present indicate that most of the seeds were found spherical followed by ovate and elliptical in shape with smooth surface and showed terminal hilum. Almost reticulate seed patterns were observed in seeds. Majority of seeds showed raised anticlinal walls with protuberance periclinal walls. The seeds of *Xanthium strumarium* were observed with maximum length of 13 mm and with width of 8 mm. Length by width ratio of seeds was also calculated; it was found that maximum L/W ratio was observed in *Sonchus oleraceus* L., i.e., 2.66. Seed characters, both macro- and micromorphological, furnish useful data for classification and delimitation of invasive taxa. This study will help to understand the invasion mechanism in plants due to variations in seed surface, shape, and other characters. Adaptive behavior of the seed during the invasion process of the new ecosystem is also elaborated.

## 1. Introduction

Invasive plant species are species that are exotic to an ecosystem. They are aggressive in nature and adversely affect ecosystems and biodiversity. They also have negative effects on the environment and cause harm to the economy and human health as well [1]. Biological invasion can lead to alterations in species composition and changes in nutrient cyclic and result in forest fire [2]. In Pakistan, alien invasive plants are considered as one of the biggest and neglected hazards to the native biodiversity [3]. The climatic characteristics like temperature, day length, and relative humidity act as an abiotic filter for newly introduced plants [4]. A study by [5] has also shown that there is no significant relationship between heat waves and alien plant species.

Exotic plant species which invade successfully have strong reproduction capacity such as higher rate of seed production, short life cycle, better seed dispersal, and germinate faster; for example, one ragweed has a capacity of production of 2000-8000 seeds [6]. Invasive plant species also produce seeds which are small and light weight which help them to disperse with wind easily and travel long distances [7]. For plants, seeds are a means of survival of the species as they carry the parent germplasm and protected against heat, cold, drought, and water. Invasive plants show strong environmental adaptability; when these plants arrive in a new environment, they change their morphology, genetic characters, and behavior which are helpful for their survival in the new environments. The seed coat characters are generally considered as stable and slightly affected by external environmental factors [8].

Many invasive plants reproduce through seeds, so seed traits are essential for invasive plant performance during the invasion process. The variations in seed traits such as seed size, morphology, and mass could be determined by geographical or environmental variables which include precipitation and temperature [9]. Seed size and mass influence the rate and speed of germination [10]. Most of the studies showed that heavier seeds have higher rate of germination due to more resource reserves [11, 12]. However, there is no significant relationship between seed mass and germination [13].

The seed coat characters can be used successfully to resolve phylogenetic and systematic problems among the taxa. In the current study, the macro- and micromorphological characters of seeds of invasive plants of Lesser Himalayas, including seed shape, size, surface, seed inner color, position of hilum, compression, length, width, and L/W ratio were observed using LM and SEM. Most taxonomists agree that data concerning the macro- and microstructure of seeds are very significant for the classification and correct identification of species. The micromorphology and ultrastructural data have contributed useful information for the evolution and classification of seed plants and play a significant role in modern synthetic systems of angiosperms [14]. Seed characters are essential to separate among genera and species of plants. The characters such as shape, color, and size of the seed are helpful in correct identification.

Scanning electron microscopy is an innovative method used to study seed ornamentation, seed molding, and evaluation of micromorphological characters of seeds that were not previously possible with light microscopy [15]. Micromorphological features of seeds along with size and shape are diagnostic tools to identify various plant species [16]. Earlier literature has also proved that seed, macro- and micromorphological features, can be used for correct identification purposes [17].

Thus, the present investigations were carried out with macro- and micromorphological (light microscopy and scanning electron microscopy) characters of seeds of 20 alien invasive plant species from Lesser Himalayas, Pakistan, to elucidate the systematic value of seed morphological characters as a criterion for separation of genera and species.

## 2. Materials and Methods

### 2.1. Sampling Area Description

The present study was carried out on the invasive plant species of Lesser Himalayas. The study area is divided into subtropical and semiarid zone with hot and humid summers from May to June while cold temperatures from October to February and from July to August; there is a monsoon season [18]. A well-developed, diverse, and abundant flora is present in this region. A variety of ornamental trees have been planted here which enhanced the beauty of this region [19]. The southern parts of Lesser Himalayas receive 70-90 mm average rainfall, while the northern parts receive 100-130 mm. A large part of the winter precipitation from the western disturbance is received in the form of snow. The northern parts receive little rain but heavy snowfall in the winter [20, 21].

### 2.2. Taxon Sampling

To obtain seeds, mature seeds of invasive plants were removed from fruits collected during field visits in the fruiting season. Seeds of some plants were purchased from herbal shops.

### 2.3. Light Microscopic Analysis of Seeds

Mature seeds of invasive plants were passed through an ethanol series (60-80%) for 1 to 3 minutes to remove the debris present on the surface. External color, shape, size (length and width), and hilum were observed using binocular dissecting microscope, placed in Plant Anatomy Lab Department of Plant Sciences in the Quaid-i-Azam University, Islamabad, Pakistan.

### 2.4. Scanning Electron Microscopic Analysis of Seeds

For SEM, seeds were immersed in absolute ethanol and left for a minute for drying. This step was carried out for a finer and detailed study of seeds. Then, the seeds were mounted on stubs in different positions, and gold coating was performed in the sputtering chamber using SPI-MODEL™. In all cases, seeds of at least 10 samples of each species were analyzed, characterized, and photographed with a scanning electron microscope (Model JEOL JSM-5910). The following seed characters were observed: the length of surface sculpture and anticlinal and periclinal wall.

## 3. Results and Discussion

In the current study, seed coat morphology of twenty seeds of invasive plant was studied, i.e., *Ailanthus altissima*, *Argemone ochroleuca*, *Azadirachta indica*, *Calotropis procera*, *Cannabis sativa*, *Cassia occidentalis*, *Chenopodium ambrosioides*, *Datura innoxia*, *Dodonaea viscosa*, *Lantana urticoides*, *Lantana camara*, *Nasturtium officinale*, *Ricinus communis*, *Robinia pseudoacacia*, *Sapium sebiferum*, *Sesamum indicum*, *Silybum marianum*, *Solanum surattense*, *Sonchus oleraceus*, and *Xanthium strumarium* (Table 1). The dominant seed was spheroidal followed by obovate and elliptical. Seeds of 12 invasive plants were found with smooth surface followed by 6 with rough surface and with ridges and furrows followed by single invasive plant species. As far as the position of hilum is concerned, 15 invasive plants showed terminal, while in 5 plants, it was not clear. The seed of *Xanthium strumarium* was observed with a maximum length of 13 mm to width of 8 mm. Length to width ratio of seeds was also calculated, and it was found that the maximum L/W ratio was observed in *Sonchus oleraceus*, i.e., 2.66 (Table 2 and Figure 1).

### 3.1. *Ailanthus altissima* (Mill.) Swingle

*Ailanthus altissima* is placed in the family Simaroubaceae, which comprises of 32 genera and more than 170 species. Brownish color seeds with light brown internal color was noted in *Ailanthus altissima*. The seed shape was spherical globose and the texture was smooth. The compression was lateral, while the hilum was not visible in the seeds. The length of the seed was 8 mm, whereas the width of the seeds was 6.5 mm, while length to width ratio of 1.2 was recorded. Figures 2(a) and 3(a) represent the SEM results of *Ailanthus altissima* that indicates smooth seed sculpturing with protruding periclinal walls. The morphological variation of the seeds seems to reflect the geographical distribution of taxa, but adaptation may have played an important evolutionary role. Numerous research studies are conducted to investigate the macro- and micromorphological characteristics of seeds. *Ailanthus* is considered as highly invasive, and there are a number of characteristics which are associated with its invasiveness such as it can produce up to 300,000 anemochorous seeds [22]. The seeds of this plant have the capability of germinating in a verity of habitats and in soil conditions as well [23], and *Ailanthus s*eeds have high germination rates in disturbed environments [24].

### 3.2. *Argemone ochroleuca* Sweet, Brit. Fl. Gard

The *A. ochroleuca* belongs to the family Papaveraceae and is native to Mexico, West India, Bulgaria, Spain, Pakistan, African countries, and Europe. Golden yellow color and creamy white internal color were observed in seeds. Seeds were obovate with smooth texture. The compression was absent, while the hilum was not visible. The length of the seed was 4.5 mm, whereas the width of the seeds is 2.5 mm. On the basis of length and width measurements, the length to width ratio of 1.8 was recorded. Seed sculpturing was smooth without any projections with a flat to concave or slightly convex periclinal wall observed in *A. ochroleuca* (Figures 2(b) and 3(b)) [25]. A numerical analysis based on seed morphology of 14 taxa belonging to the family Papaveraceae was carried. The findings revealed that in *Argemone* species, the seeds were noncompressed and dark brown in color with reticulate surface and basal hilum, which is slightly different from the present study [26]. Variations in seed morphology are not only helpful in correct identification, but these characters also contribute in expansion and establishment of invasive species.

### 3.3. *Azadirachta indica* A. Juss

In *Azadirachta indica*, oblong, grey color with copper brown internal color seeds were observed. The seed texture had ridges. The lateral compression of terminal hilum was noted. The length of the seed was 9 mm, whereas the width of the seeds was 3.5 mm, while length to width ratio of 2.57 was recorded. The seeds of *A. indica* were observed using SEM, and a surface with irregular reticulate ridges was noted (Figures 2(c) and 3(c)). [27] obtained similar findings in this plant species while studying the role of trees in climate change and their authentication through scanning electron microscopy.

### 3.4. *Calotropis procera* (Aiton) Dryand

The brown seeds in *Calotropis procera* were observed, while internal color of seeds was light brown. The seed shaped was flat, broadly ovate. The seed texture was smooth. The compression was dorsoventral, while the hilum was terminal and was observed in the seeds. The length of the seed was 5.5 mm, whereas the width of the seeds was 4.5 mm. On the basis of length and width measurements, a length to width ratio of 1.2 was recorded. Micromorphology characteristics of the seeds were studied using SEM, and the results indicated that the surface of the seed was striate ornamentation with irregular arranged granule like structures and tiny apertures. Anticlinal walls were smooth and thin, while periclinal walls were raised with thick irregular cell arrangement (Figures 2(d) and 3(d)). [28] found similar seed sculpturing in species of *Calotropis.* Seed morphology and seed coat anatomy were studied by [29] in some species of Apocynaceae and Asclepiadeceae using LM and SEM and found that the potential taxonomic value of the recorded characters is indicated by the richness of variation recorded in the sample of genera and species. He also investigated the seeds of *Calotropis procera* with hairy texture and papillate coat that is contrary to the present results. The microstructure of seeds provides data that is useful for the determination of various environmental factors on the phenotypic variability of species.

### 3.5. *Cannabis sativa* L.

*Cannabis sativa* of Cannabaceae is considered as a highly noxious weed. In the present study, the greyish brown seeds with creamy white internal color was observed. The seed shape was oblong. The seed texture was smooth. The compression was lateral, while the hilum was terminal and was observed in the seed. The length of the seed was 5.5 mm, whereas the width of the seeds was 3-4 (3.5 mm), while length to width ratio of 1.57 was recorded. Seeds were analyzed using SEM, and the findings showed that the seed surface pattern was smooth but more or less papillate (Figures 2(e) and 3(e)). The position of the hilum was apical and almost circular; the same results were found in seeds of *C. sativa* [30].

### 3.6. *Cassia occidentalis* L.

This plant is a part of the family Fabaceae which is mostly found in South America, Brazil, and Pakistan. In the current study, it was noted that seeds were grey in color with brown internal color. The shape of the seed was ovate with smooth seed texture. The compression was lateral, while the hilum was terminal and was observed in the seeds. The length of the seed was 4.5 mm, whereas the width of the seeds was 3.5 mm, and a length to width ratio of 1.28 was recorded. Micromorphological features showed that in *Cassia occidentalis*, the seed surface pattern was reticulate with granular projections. Cell shape was crooked angular, while anticlinal wall with protrusion and periclinal wall with depressed elevation were observed (Figures 2(f) and 3(f)). Our results correlate with the findings of [28].

### 3.7. *Chenopodium ambrosioides* L.

Green color seeds with blackish brown internal color was noted in *Chenopodium ambrosioides.* The spherical seed with rough texture was observed. The compression was absent, while the hilum was not visible. The length of the seed was 2 mm, whereas the width of the seeds was 1.5 mm, and a length to width ratio of 1.33 was recorded. The scanning electron microscopic analysis revealed that the seed surface punctuates and was sculptured with ruminate lines (Figures 2(g) and 3(g)).

### 3.8. *Datura innoxia* Mill

*D. innoxia* is placed in the family Solanaceae, the plants of this family are widely distributed in South Western USA, South and Central America, Western India, Afghanistan, Pakistan, India, and Malaysia. The seeds were brown in color, and the internal color was creamy white. The seed shape was like a broad kidney, while seed texture was rough. The compression was dorsoventral, while the hilum was not visible. The length of the seed was 4.5 mm, whereas the width of the seeds was 3 mm, and a length to width ratio of 1.5 was recorded. Seeds of *D. innoxia* were visualized using SEM, and the results revealed that the sculpturing was smooth rough with elongated to polygonal cells. Wrinkled or ridges with small projections and dentate or slightly straight margins were observed. Deep anticlinal wall and flat to concave periclinal wall were noted in seeds of this species (Figures 2(h) and 3(h)). In *D. innoxia*, similar pattern was observed by [25].

### 3.9. *Dodonaea viscosa* (Linn.) Jacq

*Dodonaea viscosa* belongs to the family Brassicaceae. The black seed coat color with internal color was yellow observed in *Dodonaea viscosa*. The seed was spherical in shape, and the texture was smooth. The lateral compression and terminal hilum were observed in the seeds. The length of the seed was 3.5 mm, whereas the width of the seeds was 3-4 (3.5 mm). Therefore, a length to width ratio of 1 was recorded. Scanning electron microscopic investigations showed that the surface was reticulated with variously shaped depressions in succession, while the anticlinal walls were elevated. Seed coat of *Dodonaea viscosa* showed concave periclinal walls. The concave periclinal surface walls of the seed coat have also been shown in Brassicaceae [31] (Figures 2(i) and 3(i)). To distinguish the ordered contrasts in the morphology of related genera of Brassicaceae, the SEM has been used in earlier studies.

### 3.10. *Lantana urticoides* Hayek

*Lantana urticoides* is commonly known as Texas lantana, widely distributed in Central America, Pakistan, and Mexico. Brown-colored seed with light yellow internal color was noted in *Lantana urticoides*. Spheroid-ovate seed with wrinkled texture was observed. The compression was absent, while the hilum was terminal in the seeds. The length of the seed was 5 mm, whereas the width of the seeds was 4.5 mm. Therefore, length to width ratio of 1.11 was recorded. SEM results showed that the surface sculpturing was reticulated with granular projections. The cell arrangement was irregular, and the anticlinal walls were smooth and elevated, while the periclinal walls were thin, faintly raised, and flat [32] (Figures 2(j) and 3(j)).

### 3.11. *Lantana camara* L.

*Lantana camara* is an evergreen shrub commonly known as tick berry. This plant species was introduced as an ornamental plant, but now due to its vigorous growth, it became invasive. It is native to Southeast Asia, India, and Australia. The seeds were brown in color with light yellow internal color. The seed shape was spheroid-ovate, and the texture was wrinkled. The compression was absent, while the hilum was terminal. The length of the seed was 5 mm, whereas the width of the seeds was 4.5 mm. Therefore, length to width ratio of 1.11 was recorded. The seeds showed striate surface pattern with rectangular cell shape. Smooth, depressed, thick anticlinal walls and deeply groove, rough periclinal walls were noted in *L. camara* while studying micromorphology using SEM (Figures 2(k) and 3(k)). An investigation on the oil content determination and seed morphology of Verbenaceae were conducted and found similar results as in the present research study [32].

### 3.12. *Nasturtium officinale* R. Br

*Nasturtium officinale* is placed in the family Brassicaceae, which is one of the largest families in the Angiospermae, and it can be easily distinguished by its flower and fruit characteristics. It is a family of cosmopolitan plants mainly distributed in temperate zones and Mediterranean region; this family is represented by 338 genera and 3709 species [33]. The seeds were brown in color, while internal color was light yellow. Elliptical seeds with wrinkled texture was observed in *Nasturtium officinale*. The compression was dorsoventral, while the hilum was terminal. The length of the seed was 9 mm, whereas the width of the seeds was 7 mm, and a length to width ratio of 1.28 was recorded. Micromorphological analysis revealed that the cell arrangement was reticulated with well-defined outer boundaries, and the anticlinal walls were raised and straight (Figures 2(l) and 3(l)). These findings are correlated with the findings of [34]. Reticulate sculpturing in some Barbarea taxa of the family Brassicaceae was also observed by [35].

### 3.13. *Ricinus communis* L.

*Ricinus communis* belongs to the family Euphorbiaceae, a diverse family of flowering plants which are economically essential. The seeds of *Ricinus communis* were brown in color with white internal color. The seed shape was oblong, and texture was smooth. The compression was dorsoventral, while the hilum was terminal. The length of the seed was 14 mm, whereas the width of the seeds were 6 mm, and a length to width ratio of 2.33 was recorded. SEM result indicated that the seeds of *R. communis* (Figures 2(m) and 3(m)) were spherical, rough, sculpturing, asymmetrical, and with reticulate cell arrangement with minute apertures, thick anticlinal walls, and raised smooth periclinal walls. Similar findings were noted in seeds of *Ricinus communis* by [28].

### 3.14. *Robinia pseudoacacia* L.

In *Robinia pseudoacacia*, black-brown seeds with light brown internal color were observed. The seed was kidney-shaped, and texture had furrows. The compression was lateral, while the hilum was not visible. The length of the seed was 5.5 mm, whereas the width of the seeds was 4 mm. Therefore, length to width ratio of 1.37 was recorded. The seed surface pattern was regulated; [36] also observed the same seed coat pattern in this plant species (Figures 2(n) and 3(n)).

### 3.15. *Sapium sebiferum* (L.) Roxb

The seeds were white in color with brown internal color. The seeds of *Sapium sebiferum* were globular spheroid in shape, while texture was smooth (shiny). The compression was ventral, while the terminal hilum was observed. The length of the seed was 9.5 mm, whereas the width of the seeds was 6 mm. Therefore, length to width ratio of 1.58 was recorded. Smooth seed surfaces with reticulate sculpturing with protruding periclinal walls were studied via SEM (Figures 2(o) and 3(o)). In 2015, [37] studied the reticulate seed surface pattern in some Euphorbia taxa distributed in Turkey.

### 3.16. *Sesamum indicum* L.

In *Sesamum indicum*, a grey seed coat with white internal color was noted. The obovate seed shape was with smooth (shiny) texture observed in *Sesamum indicum.* The compression was lateral, while the hilum was terminal. The length of the seed was 4.5 mm, whereas the width of the seeds was 3 mm. Therefore, a length to width ratio of 1 was recorded. Seed coat (testa) texture varied from reticulately rough to smooth at two extremes. Reticulate seed surface in *S. indicum* was also observed by [38] (Figures 2(p) and 3(p)).

### 3.17. *Silybum marianum* (L.) Gaertn

The grey seeds with internal white color were observed in *Silybum marianum*. The seed shape was oblong, and the seed texture was smooth (shiny). The dorsoventral compression terminal hilum was observed in the seeds. The length of the seed was 6 mm, whereas the width of the seeds was 2.5 mm, and length to width ratio of 2.4 was recorded. Micromorphology analysis showed that the seed surface was reticulate rugose; thin raised anticlinal cells were observed (Figures 2(q) and 3(q)), while smooth and convex periclinal walls were noted in *Silybum marianum* by [39].

### 3.18. *Solanum surattense* Burm. f

*S. surattense* belongs to the family Solanaceae which is one of the most important and large families of flowering plants. The family is widely distributed in a diversity range of ecological habitats in both tropical and temperate regions. It consists of about 98 genera and 2700 species [40]. The seeds of *S. surattense* were brown-orange in color with yellow internal color. Discoid obovate-shaped seeds with smooth (shiny) texture were observed. The compression was lateral, while the hilum was terminal. The length of the seed was 3.5 mm, whereas the width of the seeds was 2.25 mm, and a length to width ratio of 1.55was recorded. Ridged with irregular and reticulate surface was noted in the seed surface (Figures 2(r) and 3(r)). Reticulate irregular surface in the seed coat of native and naturalized species of *Solanum* was noted by [41, 42].

### 3.19. *Sonchus oleraceus* L.

*S. oleraceus* belongs to the Asteraceae family. The dark brown seeds with creamy white internal color were noted in this invasive species. The seed shape was ovate, while smooth texture was observed. The compression was dorsoventral, while the hilum was terminal. The length of the seed was 4 mm, whereas the width of the seed was 1.5 mm, and length to width ratio of 2.66 was recorded. The SEM results showed that seed surface was reticulate and anticlinal walls were thin, wavy, and grooved, while the periclinal walls were striated and grooved (Figures 2(s) and 3(s)). These results match with the findings of [39].

### 3.20. *Xanthium strumarium* L.

*X. strumarium* belongs to Asteraceae family. In this invasive species, brownish seeds with internal grey color were observed. The seed shape was oblong ellipsoid, and seed texture was rough (spiny). The compression was dorsoventral, while the hilum was terminal. The length of the seed was 13 mm, whereas the width of the seeds was 8 mm. On the basis of measurements of length and width, the length to width ratio of 1.625 mm was recorded. Scanning electron microscopy results indicated that the seed surface was spiny and rough with tetra to polygonal anticlinal cell walls, while shallow periclinal walls were observed (Figures 2(t) and 3(t)).

## 4. Conclusion

From the above results, it can be seen that a clear cut distinction can be made between taxa based on the main external morphology of seeds. Seed morphological characters provide an aid in distinguishing various species and support their placement in different clades [43]. The present study indicates that the use of seed morphological characters is a useful parameter for species identification in invasive plants. In addition to the morphological characters of seeds, texture and sculpturing of features of the external seed coat show variations among species and can be proved essential systematically [44]. The micromorphological characteristics of seeds using scanning electron microscope have been used to identify and distinguish species [45]. It can be concluded from the findings of the current studies that macro- and micromorphological characteristics of seeds are considered diagnostic at both generic and specific level of invasive plant species among the wide range of taxa. We recommend that future studies on invasive plants with special reference to macro- and micromorphological characters of seeds will provide a new perspective for understanding the invasion process.

## Figures and Tables

**Figure 1:** L/W ratio of seeds of invasive plant species of Lesser Himalaya Pakistan.

**Figure 2:** General seed view. (a) Ailanthus altissima, (b) Argemone ochroleuca, (c) Azadirachta indica, (d) Calotropis procera, (e) Cannabis sativa, (f) Cassia occidentalis, (g) Chenopodium ambrosioides, (h) Datura innoxia, (i) Dodonaea viscosa, (j) Lantana urticoides, (k) Lantana camara, (l) Nasturtium officinale, (m) Ricinus communis, (n) Robinia pseudoacacia, (o) Sapium sebiferum, (p) Sesamum indicum, (q) Silybum marianum, (r) Solanum surattense, (s) Sonchus oleraceus, and (t) Xanthium strumarium.

**Figure 3:** Seed surface view. (a) Ailanthus altissima, (b) Argemone ochroleuca, (c) Azadirachta indica, (d) Calotropis procera, (e) Cannabis sativa, (f) Cassia occidentalis, (g) Chenopodium ambrosioides, (h) Datura innoxia, (i) Dodonaea viscosa, (j) Lantana urticoides, (k) Lantana camara, (l) Nasturtium officinale, (m) Ricinus communis, (n) Robinia pseudoacacia, (o) Sapium sebiferum, (p) Sesamum indicum, (q) Silybum marianum, (r) Solanum surattense, (s) Sonchus oleraceus, and (t) Xanthium strumarium.

**Table 1:** Checklist of invasive plant species with collection site.

S. no.	Taxa	Family	Locality in Lesser Himalaya	Coordinates	Voucher specimen no.
1	*Ailanthus altissima*	Simaroubaceae	Margalla Hills	33°44′51.55^″^N 73°08′13.95^″^E	IAS-18
2	*Argemone ochroleuca*	Papaveraceae	Damn-e-Koh	33°44′38.00^″^N 73°01′22.00^″^E	IAS-02
3	*Azadirachta indica*	Meliaceae	Islamabad (Chak Shahzad)	31° 2′14.01^″^N 73° 4′32.18^″^E	IAS-08
4	*Calotropis procera*	Apocynaceae	QAU Colony	33°44′44.71^″^N 73°9′26.55^″^E	IAS-10
6	*Cannabis sativa*	Cannabaceae	QAU Isb	33°45′40.28^″^N 73°08′03.95^″^E	IAS-07
6	*Cassia occidentalis*	Fabaceae	Margalla hills (Rumli Village)	33°44′51.55^″^N 73°08′13.95^″^E	IAS-06
7	*Chenopodium ambrosioides*	Amaranthaceae	Damn-e-Koh	33°44′38.00^″^N 73°01′22.00^″^E	IAS-21
8	*Datura innoxia*	Asteraceae	QAU Isb	33°45′40.28^″^N 73°08′03.95^″^E	IAS-19
9	*Dodonaea viscosa*	Spindaceae	Margalla Hills	33°44′51.55^″^N 73°08′13.95^″^E	IAS-09
10	*Lantana urticoides*	Verbenaceae	Damn-e-Koh	33°44′38.00^″^N 73°01′22.00^″^E	IAS-17
11	*Lantana camara*	Verbenaceae	Margalla Hills	33°44′51.55^″^N 73°08′13.95^″^E	IAS-13
12	*Nasturtium officinale*	Brassicaceae	Murree road	33°44′38.00^″^N 73°01′22.00^″^E	IAS-03
13	*Ricinus communis*	Euphorbiaceae	QAU Isb (near Quaidian hut)	33°45′40.28^″^N 73°08′03.95^″^E	IAS-11
14	*Robinia pseudoacacia*	Fabaceae	Islamabad (H8)	30°44′58.73^″^N 73°12′37.27^″^E	IAS-01
15	*Sapium sebiferum*	Euphorbiaceae	Islamabad (H8)	30°44′58.73^″^N 73°12′37.27^″^E	IAS-16
16	*Sesamum indicum*	Pedaliaceae	Murree road	33°44′38.00^″^N 73°01′22.00^″^E	IAS-04
17	*Silybum marianum*	Asteraceae	Social hut QAU	33.4457° N 73.0814° E	IAS-20
18	*Solanum surattense*	Solanaceae	Margalla Hills	33°44′51.55^″^N 73°08′13.95^″^E	IAS-14
19	*Sonchus oleraceus*	Asteraceae	Chemistry hut parking, QAU	33.4446° N 73.0759° E	IAS-05
20	*Xanthium strumarium*	Asteraceae	Chemistry hut, QAU	33.4447° N 78.0804° E	IAS-12

**Table 2:** Seed macro- and micromorphological traits of invasive plant species of Lesser Himalayas Pakistan.

Sr. no.	Plant name	Seed color	Inner color	Seed shape	Texture/surface	Hilum	Compression	Length (mm)	Width (mm)	L/W ratio
1	*Ailanthus altissima*	Brown	Light brown	Spherical globose	Smooth	Not visible	Lateral	7-9 (8)	5-8 (6.5)	1.23
2	*Argemone ochroleuca*	Golden yellow	Off-white	Obovate	Smooth	Not visible	Absent	4-5 (4.5)	2-3 (2.5)	1.8
3	*Azadirachta indica*	Grey	Copper brown	Oblong	Ridges	Terminal	Lateral	8-10 (9)	3-4 (3.5)	2.57
4	*Calotropis procera*	Brown	Light brown	Flat, broadly ovate	Smooth	Terminal	Dorsoventral	5-6 (5.5)	4-5 (4.5)	1.2
5	*Cannabis sativa*	Greyish brown	Off-white	Oblong	Smooth	Terminal	Lateral	5-6 (5.5)	3-4 (3.5)	1.57
6	*Cassia occidentalis*	Grey	Brown	Ovate	Smooth	Terminal	Lateral	4-5 (4.5)	3-4 (3.5)	1.28
7	*Chenopodium ambrosioides*	Green	Blackish brown	Spherical	Rough	Not visible	Absent	1-3 (2)	0.5-2.5 (1.5)	1.33
8	*Datura innoxia*	Brown	Off –white, creamy	Broad kidney	Rough	Not visible	Dorsoventral	4-5 (4.5)	2-4 (3)	1.5
9	*Dodonaea viscosa*	Black	Yellow	Spherical	Smooth	Terminal	Lateral	3-4 (3.5)	3-4 (3.5)	1
10	*Lantana camara*	Brown	Light yellow	Spheroid-ovate	Wrinkled	Terminal	Absent	4-6 (5)	4-5 (4.5)	1.11
11	*Lantana urticoides*	Brown	Light yellow	Spheroid-ovate	Wrinkled	Terminal	Absent	4-6 (5)	4-5 (4.5)	1.11
12	*Nasturtium officinale*	Brown	Light yellow	Elliptical	Wrinkled	Terminal	Dorsoventral	8-10 (9)	6-8 (7)	1.28
13	*Ricinus communis*	Brown	White	Oblong	Smooth	Terminal	Dorsoventral	13-15 (14)	5-7 (6)	2.33
14	*Robinia pseudoacacia*	Brown to black	Light brown	Kidney shape	Furrows	Not visible	Lateral	5-6 (5.5)	3-4 (3.5)	1.37
15	*Sapium sebiferum*	White	Brown	Globular spheroid	Smooth (shiny)	Terminal	Ventral	8-1.1 (9.5)	5-7 (6)	1.58
16	*Sesamum indicum*	Grey	White	Obovate	Smooth (shiny)	Terminal	Lateral	4-5 (4.5)	2-4 (3)	1.5
17	*Silybum marianum*	Grey	White	Oblong	Smooth(shiny)	Terminal	Dorsoventral	5-7 (6)	2-3 (2.5)	2.4
18	*Solanum surattense*	Brown-orange	Yellow	Discoid obovate	Smooth (shiny)	Terminal	Lateral	3-4 (3.5)	2-2.5 (2.25)	1.55
19	*Sonchus oleraceus*	Dark brown	Off -white	Ovate	Smooth	Terminal	Dorsoventral	3-5 (4)	1-2 (1.5)	2.66
20	*Xanthium strumarium*	Brown	Gay	Oblong ellipsoid	Rough (spiny)	Terminal	Dorsoventral	12-14 (13)	7-9 (8)	1.625

## Data Availability

The data used to support the findings of this study are included within the article.
